The article "Clinical Symptoms and Quality of Life Improvement Value of Ornidazole Mixture in Auxiliary Filling Treatment of Patients with Endodontic Disease" was published in 2022. Journal: Contrast Media Mol Imaging.

# Clinical Symptoms and Quality of Life Improvement Value of Ornidazole Mixture in Auxiliary Filling Treatment of Patients with Endodontic Disease

**DOI:** 10.1155/2022/7181258

**Published:** 2022-07-07

**Authors:** Nana Sun, Nannan Wang, Lina Qu

**Affiliations:** ^1^Department of Stomatology, Beijing Chao-Yang Hospital, Capital Medical University, Beijing, China; ^2^Department of Emergency, Beijing Chao-Yang Hospital, Capital Medical University, Beijing, China; ^3^Department of Stomatology, Guang'anmen Hospital China Academy of Chinese Medical Sciences, Beijing, China

## Abstract

To evaluate the clinical effect of ornidazole mixture in auxiliary filling of patients with endodontic disease. A total of 124 patients with endodontic diseases admitted to our hospital from January 2020 to December 2021 were included and divided into two groups according to the random number table. The observation group (*n* = 62) was given ornidazole mixture-assisted filling, while the control group (*n* = 62) was given pulp mummification filling to evaluate its application effect. Compared with the control group, the disappearance time of tooth hyperesthesia, gingival redness, and pain symptoms in the observation group were significantly shorter and the difference had statistical significance (*P* < 0.05); the excellent and good rate of the observation group was 96.77% and 85.48%, respectively, and the difference had statistical significance (*P* < 0.05); the masticatory efficiency, occlusal force, and oral health-related quality of life scores in the observation group were higher than those in the control group after treatment, and the difference had statistical significance (*P* < 0.05). Ornidazole mixture can promote the curative effect, shorten the time of symptom disappearance, and effectively improve the masticatory function and quality of life in patients with endodontic diseases.

## 1. Introduction

Endodontic disease is a common disease in the stomatology department, which is mostly caused by dental hard tissue and pulp tissue lesions. Patients may have masticatory pain, gingival redness, and swelling and can cause tooth radiation pain, increasing patients' pain and reducing their quality of lives [1]. Clinical studies have confirmed that microbial infections are the main cause of endodontic disease, with specific anaerobic bacilli and parthenogenic anaerobes being the most common [2]. Therefore, the clinical treatment of this disease is based on the principle of antibacterial therapy. It is important to note that untimely treatment of endodontic disease can lead to a prolonged course of the disease, which in the long run may cause changes in tooth color and increase the risk of gingivitis or loosening of the teeth. This can not only aggravate the disease but also make treatment much more difficult [3]. Therefore, it is necessary and urgent to treat the disease by effective measures in time.

The article "Clinical Symptoms and Quality of Life Improvement Value of Ornidazole Mixture in Auxiliary Filling Treatment of Patients with Endodontic Disease" was published in 2022. Journal: Contrast Media Mol Imaging.

In the past, conventional fillers were mostly used for permanent root canal filling in the clinical treatment of endodontic diseases. Although this treatment was able to provide some relief from pain and other symptoms, it was not able to achieve a radical cure and there was still a high probability of recurrence after treatment [4]. Ornidazole, as one of the common drugs for filling therapy in recent years, is included in the category of nitroimidazoles, which contain nitro that can be successfully reduced to amino under anaerobic conditions, thus accelerating the extinction of microorganisms and exerting significant antibacterial efficacy [5]. In this paper, we have attempted to use ornidazole combination in the treatment of endodontics as an adjunct to filling therapy and compared its effectiveness with that of dry pulp fillers.

## 2. Patients and Methods

### 2.1. Patients

A total of 124 patients with endodontic diseases admitted to the Department of Stomatology of our hospital from January 2020 to December 2021 were selected as the study subjects. They were divided into the observation group (*n* = 62) and the control group (*n* = 62) according to the random number table. There was no significant difference in general data between the two groups (*P* > 0.05) (Table 1). This study was reported to the Ethics Committee of the hospital and implemented after the approval (Approval No.: 2542021-3).

The inclusion criteria were as follows: patients who were diagnosed with endodontic diseases; patients with different degrees of tooth defects and gingival swelling and pain; patients who had no history of allergic reactions to the drugs used in the study; patients who had known the details of this study and voluntarily cooperated to sign an informed consent form. The exclusion criteria were as follows: patients with concurrent severe infectious diseases, blood system diseases, and infectious diseases; patients with severe dysfunction in the heart, liver, kidney, and other vital organs; pregnant women and lactating women; patients having mental illness or cognitive mental disorders; patients who did not cooperate with the whole process of research.

### 2.2. Methods

Both groups were treated routinely, with routine disinfection of the root canals and intensive anti-infection treatment. The residual carious tissue and food residue in the dentin were thoroughly removed. In the control group, on the basis of this treatment, the patient was treated with dry pulp filler, by using the formaldehyde cresol solution (GYZZ H31022710) manufactured by Shanghai ErMed Zhangjiang Biomaterials Co. (Shanghai, China). The patient was then treated with a dry pulp paste from the same manufacturer (GYZZ H31022783) for permanent filling.

The article "Clinical Symptoms and Quality of Life Improvement Value of Ornidazole Mixture in Auxiliary Filling Treatment of Patients with Endodontic Disease" was published in 2022. Journal: Contrast Media Mol Imaging.

The experimental group was treated with adjuvant filling through ornidazole combination. The treatment was carried out as follows: we chose ornidazole sodium chloride injection (State Drug Administration H20041834) manufactured by Shaanxi Jinyu Pharmaceutical Co., Ltd. (Xi'an, China) with a specification of 100 ml each, and the ratio of ornidazole to sodium chloride was 0.125 g : 0.825 g. The solution was injected into the camphorated phenol cotton balls, and the patient was treated with a temporary seal. The interval between drug changes was also 5 days/time, and the number of treatments ranged from 1 to 5 times until the patient's pain and other symptoms of pulpitis have completely disappeared. A quantity of clove oil mucoadhesive powder was selected and mixed well with the ornidazole combination until a paste-like filling was formed, and the patient was treated with a permanent filling. Both the groups were followed up for 3 months after completion of treatment.

### 2.3. Outcome Measures

We analyzed the following indications: (1) The disappearance time of tooth hyperesthesia, gingival redness, and swelling, as well as pain symptoms, were compared between the two groups. (2) The patient's masticatory efficiency and occlusal strength were evaluated before and 3 months after the treatment. The patient was instructed to chew the peanut rice freely with both teeth without swallowing and spit out all the peanut rice after 30 seconds. The patient repeats this process for a total of 3 times at 5 minutes each time. After each process, a 2 mm diameter sieve was taken, the residue in the beaker was poured into the sieve and rinsed slowly with tap water for 20 seconds, the large peanut rice residue left on the sieve was wrapped in gauze and dried and weighed, and the residue was averaged from the final weight of the three samples. The mastication efficiency was calculated as follows: mastication efficiency = (total − residue)/total × 100%. The bite force was tested by using a Tee-Tester dental bite force tester. The patient was guided to first keep the mouth naturally closed, after which the patient clenched in a staggered position with the tips of the teeth until slight discomfort occurred, and the process was maintained for 3 s. The process was repeated again after 10 s. The processes were tested for a total of 3 times, and the final bite force value was taken as the average of the three test results. (3) The patient's recovery status after the treatment was observed, and the efficacy was judged [6]. Excellent: the symptoms associated with endodontic disease disappeared completely after the treatment, the masticatory function was completely restored, the patient's alveolar bone and root tip were confirmed to be free of abnormalities by X-ray examination, and the patient was satisfied with the appearance of the teeth; good: the symptoms associated with endodontic disease disappeared mostly after treatment, the masticatory function improved substantially, the patient was still found to have some tooth, and the patient was basically satisfied with the appearance of the teeth; poor: after treatment, the patient's symptoms were not relieved or even aggravated, there was still obvious masticatory dysfunction, X-ray examination showed that there was serious alveolar bone resorption or root canal lesions, and the patient was not satisfied with the appearance of the teeth. The treatment excellent rate was calculated as follows: treatment excellent rate = (excellent + good)/total × 100%. (4) The oral health impact profile (OHIP) [7] was used to evaluate and compare the quality of life of the two groups before treatment and 3 months after the treatment. The main contents of the scale included oral pain, physical function, psychological status, and independent ability, with 14 items. The scores of all items were between 0 and 4 points. The total score was 0 to 56 points. The score was inversely proportional to the oral health-related quality of life. The score 0 meant the worse quality of life.

The article "Clinical Symptoms and Quality of Life Improvement Value of Ornidazole Mixture in Auxiliary Filling Treatment of Patients with Endodontic Disease" was published in 2022. Journal: Contrast Media Mol Imaging.

### 2.4. Statistical Analysis

In this study, Statistical Product and Service Solutions (SPSS) 25.0 software (IBM, Armonk, NY, USA) was used as a statistical analysis tool and the enumeration data were described in the form of n%. The *χ*2 test was performed, the rank sum test was used for the grade data, and the measurement data were analyzed by (*x̅* ± *s*) and were expressed; the *t*-test was used, and *P* < 0.05 was considered statistically significant.

## 3. Results

### 3.1. Time to Disappearance of Symptoms in the Two Groups

The disappearance time of all symptoms in the observation group was significantly higher than that in the control group, and there were significant differences between the two groups (*P* < 0.05), as shown in Table 2.

### 3.2. Excellent and Good Rate between the Two Groups

The excellent and good rate of treatment was higher in the observation group than in the control group, and there was significant differences between the two groups (*P* < 0.05), as shown in Table 3.

### 3.3. Masticatory Efficiency and Bite Force in Both Groups

There was no significant difference in masticatory efficiency and occlusal force before treatment between the two groups (*P* > 0.05); however, compared with that before treatment, the masticatory efficiency and occlusal force after treatment in both groups were significantly improved and the observation group had visible significant differences (*P* < 0.05) (Table 4).

The article "Clinical Symptoms and Quality of Life Improvement Value of Ornidazole Mixture in Auxiliary Filling Treatment of Patients with Endodontic Disease" was published in 2022. Journal: Contrast Media Mol Imaging.

### 3.4. Oral Health-Related Quality of Life between the Two Groups

There was no significant difference in all oral health-related quality of life scores between the two groups before treatment (*P* > 0.05); after treatment, all quality of life scores in the two groups were significantly increased, and compared with the control group, the score in the observation group was significantly higher, and the difference was significant (*P* < 0.05) (Table 5).

## 4. Discussion

The main cause of endodontic disease in patients is bacterial and microbial infection. Patients may have tooth hyperesthesia, especially allergic reactions under cold and hot temperature stimulation. At the same time, it is easy to develop gingival redness, swelling, and pain. This pain can radiate to multiple parts such as behind the ears and neck, causing great pain to patients and resulting in decreased quality of life of patients [8]. Untimely treatment of endodontic diseases will not only affect the tooth aesthetics but also may lead to oral masticatory function damage and serious and even loss of masticatory function, threatening the physical and mental health of patients [9], so that patients have low self-esteem and other adverse psychological effects. Therefore, clinical treatment of the disease must pay more attention to timeliness and avoid aggravation of the disease due to untimely treatment which further increases the difficulty of treatment.

In the previous endodontic treatment, it was mostly advocated to open the pulp of the affected tooth after complete removal of the carious tissue and give temporary sealing and filling treatment. However, endodontic disease, as an inflammatory oral disease, can easily be repeatedly infected by bacteria, and disease recurrence often occurs after temporary occlusive filling treatment, which is not conducive to improving the prognosis. Although some treatments use a permanent filling modality, conventional pulp musters are used in adjuvant filling with unsatisfactory results [10]. Even though the pulp mummification used in conventional root canal filling therapy can exert the effects of fixation, dehydration, and preservation, it has a certain disinfection and antibacterial effect; however, the effect is limited [11, 12]. This study found that the observation group was treated with ornidazole mixture-assisted filling for pulpitis, the excellent and good rate of the overall treatment was higher than of the conventional pulp filling treatment, and the disappearance time of related symptoms in the observation group was significantly shorter. The reason is that the ornidazole mixture includes two drug components, iodoform and dexamethasone, in addition to ornidazole. Ornidazole is a broad-spectrum antibacterial drug commonly used in clinical practice. The nitro group contained in ornidazole can be reduced to free radicals in an anaerobic environment and can effectively bind to bacterial intracellular receptors to kill bacteria and play an antibacterial role [13]. In addition, the dexamethasone contained in this mixture belongs to a long-acting glucocorticoid, which can further catalyze the antibacterial effect of the drug, effectively inhibit the inflammatory response, and promote the timely relief of various inflammatory response symptoms in the body. Iodoform, as a preservative, can release free iodide ions and oxidize the active groups of bacterial plasma proteins to kill bacteria and also play a good preservative role [14]. The above three drug ingredients have a good antibacterial and bactericidal effect together, have a positive effect on improving the antibacterial ability of teeth, can reduce the gingival swelling and pain as well as other symptoms in a short time, and can improve the efficacy of the pulpitis.

The article "Clinical Symptoms and Quality of Life Improvement Value of Ornidazole Mixture in Auxiliary Filling Treatment of Patients with Endodontic Disease" was published in 2022. Journal: Contrast Media Mol Imaging.

This study showed that the masticatory efficiency of patients with pulpitis treated with ornidazole mixture-assisted filling was significantly improved, while the occlusal force was greatly enhanced. This is mainly because ornidazole mixture itself has antibacterial power and can seal it in the root canal and can make the drug directly contact the lesion. This can rapidly exert the efficacy, maintain a higher drug concentration, maximize its bioavailability, and have obvious advantages in shortening the time of symptom disappearance and improving the efficacy. It also naturally improves the masticatory efficiency and occlusal force after the patient's condition is improved [15]. It is worth noting that pulpitis can affect the psychological status of patients in addition to physiological effects such as oral pain and impaired masticatory function which makes them experience adverse emotions, reducing their quality of life. Therefore, the clinical treatment of the disease needs to pay attention to changes in the quality of life of patients.

In this study, after patients received ornidazole mixture adjuvant filling therapy, oral health-related quality of life scores were significantly improved and the quality of life was greatly promoted. This is mainly due to the improvement effect of the ornidazole mixture on the efficacy of patients. This therapy can help patients restore normal masticatory function, eliminate oral pain, improve tooth aesthetics, regulate their psychological status, and ultimately promote the improvement of the overall quality of life of patients.

The article "Clinical Symptoms and Quality of Life Improvement Value of Ornidazole Mixture in Auxiliary Filling Treatment of Patients with Endodontic Disease" was published in 2022. Journal: Contrast Media Mol Imaging.

## 5. Conclusion

In summary, auxiliary filling with ornidazole mixture in the treatment of endodontic diseases helps to further improve the excellent and good rate of treatment, accelerate the disappearance of symptoms, promote the recovery of masticatory function, and effectively improve their quality of life.

## Figures and Tables

**Table 1:** Basic data of the two groups.

Group	Gender (case)		Age (years)		Disease course (day)	
	Male	Female	Span	Mean age	Span	Mean disease duration
Observation group (*n* = 62)	31	31	26 to 69	42.05 ± 5.23	1 to 6	3.52 ± 1.03
Control group (*n* = 62)	32	30	27 to 70	42.58 ± 5.30	1 to 7	3.55 ± 1.11
Χ^2^/*t*	0.032			0.561		0.156
*P*	0.857			0.576		0.876

**Table 2:** Time to disappearance of symptoms in both groups (*d*, (*x̅* ±  *s*)).

Group	Tooth hyperesthesia	Gingival redness	Pain symptom
Observation group (*n* = 62)	8.25 ± 2.86	7.02 ± 1.03	8.85 ± 2.93
Control group (*n* = 62)	12.54 ± 3.09	10.52 ± 2.20	13.51 ± 3.55
*t*	8.023	11.345	7.972
*P*	<0.001	<0.001	<0.001

**Table 3:** Comparison of excellent and good rate between the two groups ((*n*)%).

Group	Superior	Good	Poor	Overall good rate
Observation group (*n* = 62)	40 (64.52)	20 (32.26)	2 (3.23)	60 (96.77)
Control group (*n* = 62)	30 (48.39)	23 (37.10)	9 (14.52)	53 (85.48)
*Z*/*χ*^2^	2.136			4.888
*P*	0.033			0.027

**Table 4:** The masticatory efficiency with bite force in both groups (*x̅* ± *s*).

Group	Chewing efficiency (%)		*t*	*P*	Bite force (N)		*t*	*P*
	Before treatment	3 months after treatment			Before treatment	3 months after treatment		
Observation group (*n* = 62)	68.80 ± 4.02	93.54 ± 5.03	30.253	<0.001	96.65 ± 3.54	145.33 ± 8.20	42.916	<0.001
Control group (*n* = 62)	69.01 ± 4.25	80.32 ± 4.63	14.170	<0.001	96.80 ± 3.61	121.85 ± 7.09	24.791	<0.001
*t*	0.283	15.226			0.234	17.055		
*P*	0.778	<0.001			0.816	<0.001		

**Table 5:** Oral health-related quality of life scores in the two groups (points, (*x̅* ±  *s*)).

Group	Oral pain		*t*	*P*	Psychological state		*t*	*P*
	Before treatment	After treatment			Before treatment	After treatment		
Observation group (*n* = 62)	9.52 ± 2.06	2.26 ± 0.56	26.778	<0.001	6.45 ± 2.08	2.88 ± 0.85	12.510	<0.001
Control group (*n* = 62)	9.64 ± 2.25	5.84 ± 1.03	12.092	<0.001	6.51 ± 2.12	4.80 ± 1.46	5.231	<0.001
t	0.310	24.044			0.159	8.949		
P	0.757	<0.001			0.874	<0.001		

Group	Body function		*t*	*P*	Independent ability		*t*	*P*
	Before treatment	After treatment			Before treatment	After treatment		
Observation group (*n* = 62)	7.32 ± 2.63	3.40 ± 0.52	11.513	<0.001	7.98 ± 2.60	4.53 ± 1.04	9.701	<0.001
Control group (*n* = 62)	7.37 ± 2.70	5.89 ± 1.59	3.719	<0.001	8.02 ± 2.93	6.24 ± 1.82	4.063	<0.001
*t*	0.105	11.720			0.080	6.423		
*P*	0.917	<0.001			0.936	<0.001		

The article "Clinical Symptoms and Quality of Life Improvement Value of Ornidazole Mixture in Auxiliary Filling Treatment of Patients with Endodontic Disease" was published in 2022. Journal: Contrast Media Mol Imaging.

## Data Availability

The datasets used and analyzed during the current study are available from the corresponding author on reasonable request.
